The article "Synthesis of Zinc Oxide (ZnO)-Titanium Dioxide (TiO2)-Chitosan-Farnesol Nanocomposites and Assessment of Their Anticancer Potential in Human Leukemic MOLT-4 Cell Line" was retracted in 2024. Reasons: signs of a paper mill; suspected computer-generated content; unreliable results or conclusions; concerns about the data.

# Synthesis of Zinc Oxide (ZnO)-Titanium Dioxide (TiO_2_)-Chitosan-Farnesol Nanocomposites and Assessment of Their Anticancer Potential in Human Leukemic MOLT-4 Cell Line

**DOI:** 10.1155/2022/5949086

**Published:** 2022-09-28

**Authors:** Abozer Y. Elderdery, Badr Alzahrani, Siddiqa M. A. Hamza, Gomaa Mostafa-Hedeab, Pooi Ling Mok, Suresh Kumar Subbiah

**Affiliations:** ^1^Department of Clinical Laboratory Sciences, College of Applied Medical Sciences, Jouf University, Sakaka, Saudi Arabia; ^2^Faculty of Medicine, Department of Pathology, Umm Alqura University Algunfuda, Mecca, Saudi Arabia; ^3^Pharmacology & Therapeutic Department, Medical College, Jouf University, Sakaka, Saudi Arabia; ^4^Department of Biomedical Sciences, Faculty of Medicine & Health Sciences, University Putra Malaysia, 43400 UPM Serdang, Selangor, Malaysia; ^5^Centre for Materials Engineering and Regenerative Medicine, Bharath Institute of Higher Education and Research, Chennai, India

## Abstract

Leukemia is the most prevalent cancer in children and one of the most common and deadly cancers that affect adults. Several metal oxide nanoparticles, biopolymers, and phytochemicals have been discovered to target cancer cells selectively while inflicting low to no damage to healthy cells. Among the existing nanoparticle synthesis methodologies, biologically synthesized nanoparticles using phytochemicals have emerged as a straightforward, economical, and environmentally sound strategy. The synergistic antitumor potential of ZnO-TiO_2_-chitosan-farnesol nanocomposites (NCs) against leukemia MOLT-4 cells was investigated in the current study. After synthesizing the NCs, characterization of the same was carried out using XRD, DLS, FESEM, TEM, PL, EDX, and FTIR spectroscopy. To analyze its anticancer activity, MOLT-4 cells were cultured and treated at diverse dosages of NCs. The cell viability upon treatment was examined by MTT assay. The morphological and nuclear modifications were observed by dual staining. ROS and MMP levels were observed by DCFH-DA staining and Rh-123 dye, respectively. Furthermore, the caspase 3, 8, and 9 levels were examined by performing ELISA. The XRD patterns exhibited a hexagonal structure of the NCs. In the DLS spectrum, the hydrodynamic diameter of the NCs was observed to be 126.2 nm. The electrostatic interface between the ZnO-TiO_2_-chitosan-farnesol NCs was confirmed by the FTIR spectra. A significant loss of cell viability in a dosage-dependent trend confirmed the cytotoxic effect of the NCs. An elevated ROS level and MMP depletion suggested apoptosis-associated cell death via the intrinsic pathway, which was confirmed by elevated expressions of caspase 3, 8, and 9 markers. Thus, the results showed that the synthesized NCs demonstrated a remarkable anticancer potential against leukemic cells and can be potentially valuable in cancer treatments. The findings from this study conclude that this is a new approach for modifying the physicochemical characteristics of ZnO-TiO_2_-chitosan-farnesol composites to increase their properties and synergistically exhibit anticancer properties in human leukemic cancer cells.

The article "Synthesis of Zinc Oxide (ZnO)-Titanium Dioxide (TiO2)-Chitosan-Farnesol Nanocomposites and Assessment of Their Anticancer Potential in Human Leukemic MOLT-4 Cell Line" was retracted in 2024. Reasons: signs of a paper mill; suspected computer-generated content; unreliable results or conclusions; concerns about the data.

## 1. Introduction

Leukemia is cancer of the leukocytes marked by an uncontrolled proliferation of immune cells in the blood, spleen, and bone marrow [1]. Depending on the patient's age and the hemopoietic cell lineages involved, it can be categorized as either acute or chronic leukemia [2]. Radiation, stem cell transplantation, and chemotherapy drugs are the primary treatment strategies for blood cancer [3]. However, because these therapies are intense and cause several adverse effects on the immune system, finding safer and more efficient therapeutic alternatives is warranted. The MOLT-4 T cell lines were thoroughly studied immunophenotypically and karyotypically following identification of an unusual T cell receptor gamma-chain gene rearrangement. The MOLT-4 cells were found to express CD1 and CD5 immunophenotypic markers showing thymocyte characteristics [4].

Over the last several years, nanotechnology has developed into a powerful and inventive field of research, focusing on the use of nanomaterials in fields ranging from biomedicine, drug delivery, healthcare, gene delivery, environmental science, and so on [5]. The employment of nanoparticles (NPs) in disease treatments, particularly cancer, offers the possibility of destroying cancer cells while causing minute to no damage to healthy cells and tissues. Metal nanoparticles have been demonstrated to have an efficacious impact on a variety of cancers. They are known to possess the ability to get readily distributed through the body, infiltrate the cell membranes, and trigger cytotoxicity [6, 7].

Zinc oxide (ZnO) is an interesting inorganic compound with exceptional electrical, chemical, and optical characteristics that have been used in many different applications. Furthermore, owing to their antifungal, antibacterial, anticancer, drug delivery, and antidiabetic capabilities, ZnO NPs possess immense possibilities in biological applications [8]. Titanium dioxide (TiO_2_), in addition to ZnO, is a biocompatible metal with a high surface area and mesoporous characteristics. Substantial research on the use of nano-TiO_2_ in organic degradation, dye-sensitized solar cells, glucose sensors, and specifically as a carrier for delayed and sustained drug administration have been carried out [9, 10].

The article "Synthesis of Zinc Oxide (ZnO)-Titanium Dioxide (TiO2)-Chitosan-Farnesol Nanocomposites and Assessment of Their Anticancer Potential in Human Leukemic MOLT-4 Cell Line" was retracted in 2024. Reasons: signs of a paper mill; suspected computer-generated content; unreliable results or conclusions; concerns about the data.

Synthesizing multimetallic NCs of diverse sizes and shapes is advantageous because they outperform monometallic nanoparticles in terms of specificity, functionality, and structural stability [10]. Multimetallic NPs tend to exhibit unique or greater properties when integrated, as opposed to the ones displayed by their elements [6]. Moreover, the incorporation of biopolymers such as chitosan offers additional characteristics to these synthetic NPs, including biodegradability, biocompatibility, low immunogenicity, and nontoxicity [11, 12]. A range of chitosan-based NPs has been employed for tumor-targeted drug delivery applications [13, 14].

Isoprenoids are a family of phytochemicals that could trigger apoptosis as well as ROS buildup, mitochondrial disintegration, and elevated amounts of activated caspases in several cancer cell types [15]. An example of such an isoprenoid is farnesol, a 15-carbon compound, found in orange peel, strawberries, and chamomile, as well as essential oils including lemongrass, musk, citronella, rose, tolu, cyclamen, balsam, and tuberose [16, 17].

Several reports have revealed that farnesol possesses a wide array of pharmacological characteristics, such as chemopreventative, antioxidant, anxiolytic, analgesic, anti-inflammatory, depressive, and neuroprotective actions [18–21]. These properties enable its usage for treating various conditions such as diabetes, obesity, atherosclerosis, and hyperlipidemia [22]. Furthermore, its chemoprotective action has been studied in numerous cancer types including breast tumor [23, 24], lung cancer [25], colon carcinoma [26], oral squamous cancer [27], leukemia [28], and pancreatic adenocarcinoma [29].

Examining the synergistic anticancer potential of ZnO-TiO_2_-chitosan-farnesol NCs against human ALL (MOLT-4) cells is the main goal of the current work. After synthesizing the NCs, characterization of the same was carried out using XRD, DLS, FESEM, TEM, PL, EDAX, and FTIR spectroscopy. To analyze its anticancer activity, human ALL (MOLT-4) cells were grown and administered with diverse doses of NCs. After treatment, the viability of the cells was investigated by MTT assay. AO/EtBr staining revealed morphological and nuclear changes. The levels of ROS and MMP were determined using DCFH-DA staining and Rh-123 dye, respectively. Additionally, the ELISA method was used to determine the level of caspase 3, 8, and 9 proteins in the culture supernatants.

## 2. Materials and Methods

### 2.1. Synthesis of ZnO-TiO_2_-Chitosan-Farnesol NCs

The formulation of ZnO-TiO_2_-chitosan-farnesol NCs was done via the chemical precipitation technique. 500 mg of TiO_2_ NPs was combined with 0.1 M of Zn (NO_3_)_2_. Next, 50 mL of an aqueous solution containing 1% acetic acid was used to dissolve 500 mg of chitosan. In addition, 50 mg of phytochemical farnesol was mixed with the ZnO-TiO_2_-chitosan solution. The 0.1 M of NaOH solution was mixed drop by drop in ZnO-TiO_2_-chitosan-farnesol solution, and finally, the white residue was obtained. The residue was agitated at 37°C for 3 h, and then, the obtained nanopowder was rinsed thrice with distilled water followed by ethanol solutions. The resulting solution was centrifuged at −3°C for 40 min at 15,000 rpm. The final solution was dehydrated for 2 h at 200°C and obtained NCs were kept at 4°C for further studies [30].

The article "Synthesis of Zinc Oxide (ZnO)-Titanium Dioxide (TiO2)-Chitosan-Farnesol Nanocomposites and Assessment of Their Anticancer Potential in Human Leukemic MOLT-4 Cell Line" was retracted in 2024. Reasons: signs of a paper mill; suspected computer-generated content; unreliable results or conclusions; concerns about the data.

### 2.2. Characterization of ZnO-TiO_2_-Chitosan-Farnesol NCs

The obtained ZnO-TiO_2_-chitosan-farnesol NCs were studied using the XRD (model: X'PERT PRO PANalytical). ZnO-TiO_2_-chitosan-farnesol NCs XRD results were captured in the 2*θ* range of 25°–80° using a monochromatic CuK*α* diffraction beam wavelength of 1.5406 Å. The ZnO-TiO_2_-chitosan-farnesol NCs' particle size study was conducted using the NanoPlus DLS Nano Particle Sizer and then analyzed by using a SEM (Carl Zeiss Ultra 55 FESEM) with EDAX Spectrometry (model: Inca). The morphologies of the ZnO-TiO_2_-chitosan-farnesol NCs were examined by using the TEM (Tecnai F20 model) instrument. Using a Perkin Elmer spectrometer, the FTIR spectra were captured in the 400–4000 cm^−1^ wavenumber range. Photoluminescence (PL) spectrum was taken using the Perkin Elmer-LS 14 spectrometer [31].

### 2.3. Cell Culture and Treatments

The MOLT-4 cells were acquired from ATCC, USA. The cells were maintained at 37°C and cultured in DMEM media enriched with FBS (10%) and 1% penicillin/streptomycin antibiotics in a CO_2_ incubator.

### 2.4. MTT Cytotoxicity Assay

The cytotoxicity of the NCs against MOLT-4 cells was examined as per the approach of Mosmann (1983) [32]. The cells were seeded on a 96-well plate and treated with several concentrations (10–60 *μ*g/ml) of the prepared NCs for 24 h. Posttreatment, 20 *μ*l of MTT (2.5 mg/ml) was mixed, and the solution was left for incubation for an additional 4 h. Later, the formed formazan crystals were suspended in 150 *μ*l of DMSO. A spectrophotometer was employed to determine the absorbance at 570 nm. At a 50% inhibitory concentration (IC_50_), the percentage of cell viability was noted. Cell viability was determined as a percentage value of each well absorbance compared to control cell wells. The data were obtained through triplicate assays. The morphology of cells treated with the optimum concentrations was further observed under a light microscope at 20x magnification.

The article "Synthesis of Zinc Oxide (ZnO)-Titanium Dioxide (TiO2)-Chitosan-Farnesol Nanocomposites and Assessment of Their Anticancer Potential in Human Leukemic MOLT-4 Cell Line" was retracted in 2024. Reasons: signs of a paper mill; suspected computer-generated content; unreliable results or conclusions; concerns about the data.

### 2.5. AO/EtBr Staining

To observe the impact of the NCs on apoptotic cell death, the AO/EtBr staining methods were carried out. The dual stains (AO/EtBr: 100 *μ*g/ml) were combined with the cells treated with NCs (50 and 60 *μ*g/ml) for 24 h and a coverslip was placed over to smear the dye. Then, the slides were maintained for 5 min at 37°C. Using a fluorescent microscope at a magnification of 20x, the apoptotic cells were examined using a fluorescent microscope (Labomed; USA) [33]. The microscopic pictures were obtained by three independent experiments.

### 2.6. Estimation of ROS Level in the Cell

The intracellular ROS levels were assessed by DCFH-DA staining. Inside the cell, deacetylation allows the dye to react with radicals in a quantifiable form, resulting in the dye's conversion to its fluorescent byproduct DCF. After being treated with NCs (50 and 60 *μ*g/ml) for 24 h, the cells were removed and resuspended in PBS. After that, DCFH-DA solution (10 *μ*M) was added to the suspension (2 × 10^5^ cells/ml) and left for incubation for 30 min at 37°C. The cells were then cleansed twice using PBS and then examined at 485–530 nm, the fluorescence intensity was measured spectrofluorometrically using SpectraMax® M2 (Molecular Devices; USA) [31]. The data were obtained by three independent experiments in triplicates.

### 2.7. Measurement of MMP

Mitochondrial depolarization was measured using rhodamine-123 (Rh-123), a fluorescent dye. The cells were loaded in a 6-well plate and incubated with NCs (50 and 60 *μ*g/ml) for 24 h. Following the dye addition, the suspension was maintained at 37°C for 30 min. Then, it was rinsed in 1 × PBS before being examined under a fluorescence microscope (Labomed; USA), the intensity was captured with a blue filter (450–490 nm), and the fluorescence intensity of the recorded images was examined using ImageJ software [30]. The images were obtained by three independent experiments in triplicates.

### 2.8. Measurement of Caspases 3, 8, and 9 Activities

The leukemic cells were loaded in a 6-well plate containing media and the NCs (50 and 60 *μ*g/ml) for 24 h. The supernatants were harvested and sustained at −80°C. The levels of caspase 3, 8, and 9 in the extract were examined colorimetrically using kits as per the recommended protocols of the manufacturer (Abcam, USA) [32]. The data were obtained by three independent experiments in triplicates.

### 2.9. Statistical Analysis

The findings were represented as the mean ± SD of triplicates. The SPSS program version 20 was used to assess statistical analyses. One-way ANOVA and the DMRT test were used to calculate the significance level. The results are significant if *p* < 0.05.

The article "Synthesis of Zinc Oxide (ZnO)-Titanium Dioxide (TiO2)-Chitosan-Farnesol Nanocomposites and Assessment of Their Anticancer Potential in Human Leukemic MOLT-4 Cell Line" was retracted in 2024. Reasons: signs of a paper mill; suspected computer-generated content; unreliable results or conclusions; concerns about the data.

## 3. Results

### 3.1. Synthesis and Characterization of ZnO-TiO_2_-Chitosan-Farnesol NCs

The XRD patterns of ZnO-TiO_2_-chitosan-farnesol NCs are shown in Figure 1. The ZnO appears as the dominant face at angles (2*θ*) 31.70°, 34.35°, 36.20°, 47.43°, 56.48°, 62.77°, 66.30°, 67.91°, and 69.01° with corresponding hkl values of (100), (002), (101), (102), (110), (103), (200), (112) and (201) for hexagonal wurtzite structure for ZnO, and it is matched with standard JCPDS card no. 36–1451 [34]. The TiO_2_ peaks are observed at 24.27°, 29.91°, 43.79°, and 47.43° revealing the anatase TiO_2_ phase structure (JCPDS card no: 21–1272) [35]. The peaks at 10.46° and 19.64° revealed the noncrystalline chitosan. Farnesol diffraction peaks were also discovered to be 15.77° and 16.18°. The formation of ZnO-TiO_2_-chitosan-farnesol NCs was facilitated by both steric effects and intermolecular hydrogen bonding amongst the matrixes. The Debye–Scherrer formula calculated the crystallite size of the ZnO-TiO_2_-chitosan-farnesol matrix to be 52 nm [34].

FESEM/TEM/SAED patterns were utilized to determine the surface topography of the ZnO-TiO_2_-chitosan-farnesol NCs, as illustrated in Figures 2 and 3. TEM pictures showed that farnesol (first layer) and chitosan (middle layer) were encapsulated on metal oxide (ZnO-TiO_2_) in a one-by-one layered pattern (final layer).

The hexagonal structure of ZnO-TiO_2_-chitosan-farnesol NCs was also noticeable in FESEM and TEM images. The hexagonal structure formation edge was apparent in the data (Figure 3(c)). On the top of the nanorod, the metal oxide was encapsulated with biopolymer chitosan and phytocompounds farnesol. The average particle size was 50 ± 3 nm, as determined by XRD. The creation of the ZnO hexagonal wurtzite crystalline phase in the TiO_2_, farnesol, and chitosan nanomaterials was verified by the SAED pattern (figure 3(d)). The elements of synthesized ZnO-TiO_2_-chitosan-farnesol NCs were identified by the EDAX spectrum as shown in Figure 4(a). The ZnO-TiO_2_-chitosan-farnesol NCs atomic percentages were found to be 13.58% (C), 9.53% (N), 31.76% (Zn), 9.49% (Ti), and 35.11% (O) in the ZnO-TiO_2_-chitosan-farnesol NCs.

The DLS spectra of ZnO-TiO_2_-chitosan-farnesol NCs measured 126.20 nm (Figure 4(b)). Additionally, the hydrodynamic size of the DLS particle was improved in comparison to the XRD and TEM studies since the NCs were encircled by an aqueous media. The FTIR spectra are displayed in Figure 5(a). These results confirmed that the ZnO, TiO_2_, chitosan, and farnesol various functional groups were found to be present in ZnO-TiO_2_-chitosan-farnesol samples. The characteristics of the chitosan peaks were observed at 3413 and 1634 cm^−1^, which was due to the broad spectrum of OH and -NH peaks with H bonds, indicating the amide I group (C-O stretching along with the N-H distortion mode). The carboxylic acid salt peak's COO- group was located at 1316 cm^−1^. The glucose circle C-O-C stretching vibrations were observed at 1067 cm^−1^ [36]. However, the farnesol characteristics peaks, the C-H asymmetric and symmetric stretching observed at 2914 and 2837 cm^−1^, were accredited to the carboxylate group. The C-H bending (alkane) stretch peaks were observed at 1461 and 1384 cm^−1^. However, the peaks found in ZnO-TiO_2_-Farnesol at 932 cm^−1^ and 1030 cm^−1^ were because of the C-OH bending and OH stretching, respectively, and confirmed the interactions [37]. The metal-oxygen (MO) stretching vibration such as Zn-Ti-O was observed at 724 and 485 cm^−1^ [38]. The FTIR spectrum results confirmed that farnesol has successfully interacted with chitosan, ZnO, and TiO_2_ of the ZnO-TiO_2_-chitosan-farnesol surface matrix. These interactions resulted from the ZnO-TiO_2_-chitosan-farnesol NCs' electrostatic contacts with one another.

The article "Synthesis of Zinc Oxide (ZnO)-Titanium Dioxide (TiO2)-Chitosan-Farnesol Nanocomposites and Assessment of Their Anticancer Potential in Human Leukemic MOLT-4 Cell Line" was retracted in 2024. Reasons: signs of a paper mill; suspected computer-generated content; unreliable results or conclusions; concerns about the data.

The 325 nm wavelength was used to excite the NCs.  Figure 5(b) shows the ZnO-TiO_2_-chitosan-farnesol NCs' photoluminescence spectrum. Peaks in the ZnO-TiO_2_-chitosan-farnesol NCs sample emission spectrum were found at 378 nm, 395 nm, 417 nm, 442 nm, 458 nm, 474 nm, and 510 nm, respectively. UV emissions (near band edge) were discovered at 378 nm and 395 nm as a result of the free exciton collision mechanism of radiative recombination [36]. The violet emission observed at 417 nm may be caused by an electron transfer from the surface donor to the top valence band [36]. Singly ionized Zn vacancies (V_Zn_) were represented by the three blue emission bands at 442 nm, 458 nm, and 474 nm, respectively [36]. Due to oxygen vacancies (Ovs), the green emission band was centered at 510 nm [36].

### 3.2. Impact of ZnO-TiO_2_-Chitosan-Farnesol NCs on the Cell Viability

The cytotoxic potential of the NCs on MOLT-4 cell viability is depicted in Figure 6. MOLT-4 cells administered with NCs revealed substantial cytotoxicity with the IC_50_ of 47.98 *μ*g/ml. The optical microscope was engaged to investigate the morphological alterations in MOLT-4 cells. At a dosage of 50 and 60 *μ*g/ml, NCs revealed a remarkable loss of viability and the appearance of morphological abnormalities including detachment, shrinkage, membrane blebbing, and distorted shape (Figures 6(a) and 6(b)). With increased concentrations, further morphological modifications occurred. From the IC_50_ results, two concentrations of the NCs (50 and 60 *μ*g/ml) were chosen for further studies.

The article "Synthesis of Zinc Oxide (ZnO)-Titanium Dioxide (TiO2)-Chitosan-Farnesol Nanocomposites and Assessment of Their Anticancer Potential in Human Leukemic MOLT-4 Cell Line" was retracted in 2024. Reasons: signs of a paper mill; suspected computer-generated content; unreliable results or conclusions; concerns about the data.

### 3.3. NCs Induced Cell Death via Apoptosis

The apoptosis-associated cell death in NCs-treated cells was studied using a dual AO/EtBr staining method. The control cells displayed green fluorescence stained by AO, indicating living cells without apoptosis; however, the cells exposed to the NCs exhibited yellow and orange fluorescence, signifying apoptosis, with ruptured nuclei and necrotic cells. The yellow and orange fluorescence intensity increased as the dosage of the NCs increased. As a result, the capacity of NCs to cause apoptosis in MOLT-4 cells became apparent (Figure 7).

### 3.4. Measurement of Intracellular ROS Level in Cells

The DCFH-DA staining method was executed to determine the ROS production in MOLT-4 cells subjected to two different doses of NCs (50 and 60 *μ*g/ml) and the result is depicted in Figure 8. Control cells fluoresced in a dull green color, indicating minimal ROS production. MOLT-4 cells treated with NCs (50 *μ*g/ml) displayed faint background fluorescence, but those cells treated with a higher dosage of NCs (60 *μ*g/ml) showed intense green fluorescence, indicating an elevated ROS production with increased concentration of treatment with NCs (Figure 8).

### 3.5. Measurement of MMP Level in the Cells

Rh-123 staining was used to assess the MMP level in the NCs (50 and 60 *μ*g/ml) treated MOLT-4 cells, and the outcomes are illustrated in Figure 9. The control cells were found to have intense green fluorescence, which denotes a higher MMP level. However, MOLT-4 cells treated with the NCs displayed a dull green fluorescence, indicating a depleted MMP in the cells. This finding demonstrated that NCs could lower the MMP levels in MOLT-4 cells, which also explains the elevated ROS levels (Figure 9).

### 3.6. Involvement of Caspase 3, 8, and 9 Proteins in Cell Death

The NCs administered to MOLT-4 cells displayed elevated expressions of caspase 3, 8, and 9 in comparison to the control cells (Figure 10). These findings showed that ZnO-TiO_2_-chitosan-farnesol NCs induced apoptosis in MOLT-4 cells occurred via a caspase-dependent pathway. The NCs treatment increased the expression of proapoptotic markers significantly (50 *μ*g/ml, *p* < 0.05; 60 *μ*g/ml, *p* < 0.01).

## 4. Discussion

The combination of metal nanoparticles and biopolymers has been employed for the treatment of leukemia for the past few years. Chitosan, a polysaccharide obtained from chitin deacetylation, has been utilized to synthesize metal nanoparticles as a cationic reducing agent. This application is viable because of its many biological characteristics, including biocompatibility, cancer cytotoxicity, the ability to diagnose cancer, and the ability to serve as a vehicle for the transport of drugs in cancer treatments [39, 40]. Moreover, the incorporation of phytochemicals into the nanoparticle-biopolymer combination enhances the anticancer effect [41, 42].

The article "Synthesis of Zinc Oxide (ZnO)-Titanium Dioxide (TiO2)-Chitosan-Farnesol Nanocomposites and Assessment of Their Anticancer Potential in Human Leukemic MOLT-4 Cell Line" was retracted in 2024. Reasons: signs of a paper mill; suspected computer-generated content; unreliable results or conclusions; concerns about the data.

One such isoprenoid is farnesol, which has been proven to enable the induction of cell death in several cell lines [16]. Furthermore, farnesol has been demonstrated to possess selective toxicity against tumor cells, especially leukemic cells, indicating its huge potential to be employed effectively for cancer treatment [43]. Thus, the primary goals of the current study were to synthesize, characterize, and test the anticancer effectiveness of generated ZnO-TiO_2_-chitosan-farnesol NCs against leukemic MOLT-4 cell lines.

One of the most significant techniques in nanotoxicology research is the cell toxicity study, which reveals the response of cells to any toxicant and provides information on cell survival and death rates [44]. The leukemic MOLT-4 cells treated with the synthesized NCs exhibited substantial cytotoxicity in a concentration-dependent fashion. The result is concordant with a previous study conducted with zinc oxide/titanium dioxide NCs [45, 46]. Moreover, the concentration-dependent toxicity of the NCs could be accredited to the occurrence of farnesol in the synthesized NCs. Normally, farnesol is well-known for its remarkable anticancer properties compared to ZnO and TiO_2_ [28].

To further comprehend the cell death mechanism triggered by the NCs, the AO/EtBr staining method was used to assess the morphological modification associated with apoptosis. The living (control) cells fluoresced green due to the diffusion of AO into the cellular membranes, but the treated cells turned apoptotic and fluoresced orange due to nuclear shrinkage. An earlier study conducted with ZnO/TiO_2_/Ag NCs also revealed similar observations [47]. The chromatin fragmentation that occurred in the NCs-treated cells indicated an uptake of EtBr dye, as observed with chitosan decorated silver nanoparticles in an earlier report [48]. The chitosan incorporated in the NCs contains free amine groups, which not only provide a high positive surface charge but also enable it to interact easily with the negatively charged cell membrane, contributing further to cell death by apoptosis [49].

The formation of intracellular ROS frequently results in the onset of oxidative stress that results in cell death by apoptosis [50]. The primary process of NPs toxicity is free radical production and the consequent buildup of oxidative stress [51]. Also, an increased amount of ROS generated in the treated cells is linked to the initiation of early as well as late apoptosis [52]. The current study notably showed elevated ROS generation in the NCs-treated cells in a concentration-dependent trend. Previous studies have suggested that nanoparticle treatment produces superoxide and hydroxyl radicals as well as nonradical hydrogen peroxide, which cause DNA, lipids, and protein damage, as well as cell cycle arrest [51]. According to reports, ROS production is a critical factor for inducing apoptosis [53], and that abnormally high ROS accumulation can deplete the antioxidant capacity of cells, modify cellular metabolic pathways, and alter mitochondrial functioning, resulting in cell death [54].

The article "Synthesis of Zinc Oxide (ZnO)-Titanium Dioxide (TiO2)-Chitosan-Farnesol Nanocomposites and Assessment of Their Anticancer Potential in Human Leukemic MOLT-4 Cell Line" was retracted in 2024. Reasons: signs of a paper mill; suspected computer-generated content; unreliable results or conclusions; concerns about the data.

Mitochondria are known to be the primary origin of intracellular ROS. Hence, an elevated ROS level triggers the opening up of a mitochondrial transition pore, thereby reducing the MMP and activating the caspase cascade that eventually culminates in cell death [55]. In the NCs-treated cells, a faint green fluorescence was noticed, which was attributed to the mitochondrial membrane depolarization that in turn failed to retain the Rh-123 probe. An elevated ROS level triggered the apoptotic process by promoting mitochondrial membrane depolarization, corroborating previous anticancer studies conducted with cisplatin and farnesol coencapsulated nanoparticles [15].

Apoptosis is an intricate and sophisticated process that involves an energy-dependent chain of molecular processes involving cell shrinkage, chromatin condensation, and cell disintegration [16]. Since caspase activation is the starting point in the apoptotic process, assessing their activity is a significant component of the mode of action studies. Caspases are a class of proteins that are triggered by caspase 3, which triggers apoptosis by stimulating caspase 8 and 9 [56]. The synthesized NCs substantially elevated the expression pattern of proapoptotic genes and caspase 3, 8, and -9. Our findings indicated that the cytotoxic potential of the NCs in cells was mediated by apoptosis activation, which was consistent with the elevation of ROS, deterioration of MMP levels, and increased the numbers of cells exhibiting yellow and orange fluorescence in AO/EtBr staining results. In NCs-treated cells, the augmented ROS levels decreased MMP levels, and caspase activation revealed that apoptosis was being induced through the intrinsic or mitochondrial pathway [57]. Farnesol-mediated cell death in several tumor cells has also been observed to follow the intrinsic pathway, which is concomitant with the obtained results [21, 27].

## 5. Conclusion

The synergistic anticancer potential of ZnO-TiO_2_-chitosan-farnesol NCs in MOLT-4 cells has been investigated. The cytotoxic effect of the NPs along with an elevated ROS level decreased MMP level, and increased expressions of caspase 3, 8, and 9 indicated a significant anticancer potential of the NCs. The NCs were noticed to trigger apoptosis in the leukemic cells through the upregulation of the caspase 3, 8, and 9 genes and MMP depletion. Thus, the cytotoxicity of NCs was found to be mediated by apoptotic induction via the mitochondrial pathway. Overall, our findings revealed an innovative approach for modifying the physicochemical features of ZnO-TiO_2_-chitosan-farnesol NCs to enhance their properties and synergistically exhibit anticancer properties in human leukemic cancer cells.

The article "Synthesis of Zinc Oxide (ZnO)-Titanium Dioxide (TiO2)-Chitosan-Farnesol Nanocomposites and Assessment of Their Anticancer Potential in Human Leukemic MOLT-4 Cell Line" was retracted in 2024. Reasons: signs of a paper mill; suspected computer-generated content; unreliable results or conclusions; concerns about the data.

## Figures and Tables

**Figure 1:** XRD patterns of the ZnO-TiO_2_-chitosan-farnesol NCs.

**Figure 2:** Lower (a) and higher (b) magnification FESEM image ZnO-TiO_2_-chitosan-farnesol NCs.

**Figure 3:** ZnO-TiO_2_-chitosan-farnesol NCs SAED pattern (d) in lower and higher magnification TEM images (a)–(c).

**Figure 4:** EDAX spectrum (a) and DLS spectrum (b) of ZnO-TiO_2_-chitosan-farnesol NCs.

**Figure 5:** FTIR spectrum of ZnO-TiO_2_-chitosan-farnesol NCs (a). PL spectrum of ZnO-TiO_2_-chitosan-farnesol NCs (b).

**Figure 6:** The cytotoxic effect of ZnO-TiO_2_-chitosan-farnesol NCs on MOLT-4 cells. ZnO-TiO_2_-chitosan-farnesol NCs treated in the cells for 24 hours at several concentrations, and the MTT assay employed to calculate the cell viability (a). Morphological changes in MOLT-4 cells after ZnO-TiO_2_-chitosan-farnesol NCs treatment at 50 and 60 *μ*g/ml concentration for 24 h observed under the light microscope at 20× magnification (b).

**Figure 7:** Effect of ZnO-TiO_2_-chitosan-farnesol NCs triggered apoptosis in MOLT-4 cells by AO/EtBr staining. Blood cancer cells administered with ZnO-TiO_2_-chitosan-farnesol NCs for 24 h at two concentrations (50 and 60 *μ*g/ml), stained with AO/EtBr, and observed under a fluorescence microscope (a). The fluorescence image showing control MOLT-4 cells with green fluorescence, NCs (50 *μ*g/ml) treated cells with green and yellow fluorescence, and NCs (60 *μ*g/ml) treated cells with yellow and orange fluorescence (b). The values are displayed as the mean ± SD of triplicates: ^*∗*^*p* < 0.05 vs. control; ^*∗∗*^*p* < 0.01 vs. control.

**Figure 8:** DCFH-DA staining method for examination of ZnO-TiO_2_-chitosan-farnesol NCs induced ROS level.

**Figure 9:** Staining of mitochondria using Rh-123 in human MOLT-4 cells treated with ZnO-TiO_2_-chitosan-farnesol NCs.

**Figure 10:** Effect of ZnO-TiO_2_-chitosan-farnesol NCs on caspase 3 (a), 8 (b), and 9 (c) activities in MOLT-4 cells. The cells were treated for 24 h with the NCs at the dosages of 50 and 60 *μ*g/ml. The protein status in the culture supernatant was subsequently estimated by the ELISA technique. The outcomes were displayed as the mean ± SD of triplicates: ^*∗*^*p* < 0.05 vs. control; ^*∗∗*^*p* < 0.01 vs. control.

The article "Synthesis of Zinc Oxide (ZnO)-Titanium Dioxide (TiO2)-Chitosan-Farnesol Nanocomposites and Assessment of Their Anticancer Potential in Human Leukemic MOLT-4 Cell Line" was retracted in 2024. Reasons: signs of a paper mill; suspected computer-generated content; unreliable results or conclusions; concerns about the data.

## Data Availability

The data used to support the findings of this study are available from the corresponding author upon request.
